The article "Differentiating Glioblastoma Multiforme from Brain Metastases Using Multidimensional Radiomics Features Derived from MRI and Multiple Machine Learning Models" was published in 2022. Journal: Biomed Res Int.

# Differentiating Glioblastoma Multiforme from Brain Metastases Using Multidimensional Radiomics Features Derived from MRI and Multiple Machine Learning Models

**DOI:** 10.1155/2022/2016006

**Published:** 2022-09-28

**Authors:** Salar Bijari, Amin Jahanbakhshi, Parham Hajishafiezahramini, Parviz Abdolmaleki

**Affiliations:** ^1^Department of Medical Physics, Faculty of Medical Sciences, Tarbiat Modares University, Tehran, Iran; ^2^Stem Cell and Regenerative Research Center, Iran University of Medical Sciences, Tehran, Iran; ^3^Department of Biophysics, Faculty of Biological Sciences, Tarbiat Modares University, Jalal AleAhmad, Nasr, P.O. Box 14115-111, Tehran, Iran; ^4^Department of Biophysics, Faculty of Biological Sciences, Tarbiat Modares University, Tehran, Iran

## Abstract

Due to different treatment strategies, it is extremely important to differentiate between glioblastoma multiforme (GBM) and brain metastases (MET). It often proves difficult to distinguish between GBM and MET using MRI due to their similar appearance on the imaging modalities. Surgical methods are still necessary for definitive diagnosis, despite the importance of magnetic resonance imaging in detecting, characterizing, and monitoring brain tumors. We introduced an accurate, convenient, and user-friendly method to differentiate between GBM and MET through routine MRI sequence and radiomics analyses. We collected 91 patients from one institution, including 50 with GBM and 41 with MET, which were proven pathologically. The tumors separately were segmented on all MRI images (T1-weighted imaging (T1WI), contrast-enhanced T1-weighted imaging (T1C), T2-weighted imaging (T2WI), and fluid-attenuated inversion recovery (FLAIR)) to form the volume of interest (VOI). Eight ML models and feature reduction strategies were evaluated using routine MRI sequences (T1W, T2W, T1-CE, and FLAIR) in two methods with (second model) and without wavelet transform (first model) radiomics. The optimal model was selected based on each model's accuracy, AUC-roc, and F1-score values. In this study, we have achieved the result of 0.98, 0.99, and 0.98 percent for accuracy, AUC-roc, and F1-score, respectively, which have yielded a better result than the first model. In most investigated models, there were significant improvements in the multidimensional wavelets model compared to the non-multidimensional wavelets model. Multidimensional discrete wavelet transform can analyze hidden features of the MRI from a different perspective and generate accurate features which are highly correlated with the model accuracy.

## 1. Introduction

Glioblastoma multiforme (GBM) and brain metastases (MET) are the most common malignant brain tumors in adults [1, 2]. The distinction between these two types of tumors is crucial to subsequent diagnostic and therapeutic planning [3, 4]. An accurate diagnosis of the tumor's source and extent is crucial [5, 6]. In addition, treatment strategies for these tumors differ; total en bloc resection is preferred for MET, while stereotactic radiosurgery can be used for MET less than 3 to 4 cm, whereas GBM should be treated with maximal resection followed by molecular classification and simultaneous chemoradiotherapy [7–9]. Diagnosis of GBM and MET is based on histopathology biopsy [9, 10]. It is particularly dangerous for older adults and tumors near eloquent areas [9, 10]. In routine magnetic resonance imaging (MRI), GBM and MET show peripheral edema and ring enhancement [11, 12]. Even though the two lesions had different treatment strategies, similar radiological appearances made it difficult to differentiate them. Many years of radiological research have focused on accurately distinguishing these two lesions [11, 13, 14].

The article "Differentiating Glioblastoma Multiforme from Brain Metastases Using Multidimensional Radiomics Features Derived from MRI and Multiple Machine Learning Models" was published in 2022. Journal: Biomed Res Int.

A radiomics study may provide pathophysiological insights otherwise hidden in quantitative imaging data [12]. In radiomics research, some features are used, such as size, shape, image intensity, and voxel relationships [4–8]. A wide range of problems can be solved using multidimensional wavelets [15, 16]. An effective way to reveal hidden characteristics of signals is to use discrete wavelets (DWT) [15, 16].The wavelet transform is a robust tool in signal processing, and it could provide us with deep and precise insight into the structure of the signals [15, 16].

With new machine learning algorithms (ML), radiomics analysis could be more precise, accurate, and convenient for clinical reports [1–4, 6]. Predictive model can be created based on the unique patterns found in the data by using these algorithms [6–10]. Following training, the machine can accurately identify the tumor type in a new sample and support clinical decisions significantly. In MRI images, brain tumors can be categorized in many ways [10–14]. One of the most prominent ones is fuzzy clustering means (FCM), support vector machine (SVM), artificial neural network (ANN), knowledge-based techniques, and the expectation-maximization (EM) algorithm methodology [14, 17–19].

It has been reported that advanced techniques of MRI, such as perfusion-weighted imaging (PWI), diffusion tensor imaging (DTI), MR spectroscopy (MRS), and amide proton transfer-weighted imaging, play vital roles in the diagnosis of GBMs compared with MET; however, these advanced techniques may not be included in all standard MRI protocols [3, 12, 20]. Any single finding cannot guide clinical practice in some cases due to diagnostic uncertainty. Many previous studies showed that combined conventional MRI (cMRI), diffusion-weighted imaging (DWI), and 18F-FDG-PET images to establish different radiomics models to differentiate MET from GBM and found that the integrated model based on cMRI, DWI, and 18F-FDG-PET had the best discriminatory power. In contrast, advanced sequences like DWI are not widely available in the clinic as cMRI [3, 12, 20]. Consequently, the radiomics literature shows that different classifiers have different outputs [1–6]. Choosing the best model is complex [3–6]. It is necessary to build various models to achieve a more excellent result [3, 12, 20].

The article "Differentiating Glioblastoma Multiforme from Brain Metastases Using Multidimensional Radiomics Features Derived from MRI and Multiple Machine Learning Models" was published in 2022. Journal: Biomed Res Int.

In this study, we have used standard MRI sequences (T1-weighted imaging (T1WI), contrast-enhanced T1-weighted imaging (T1C), T2-weighted imaging (T2WI), and fluid-attenuated inversion recovery (FLAIR)) to extract the features from the dataset. By combining these simple features with DWT, we developed suitable feature vectors that can be used in machine learning algorithms to differentiate between GBM and MET patients. The objective of our study was to develop a convenient, accurate, and stable predictive model to aid clinical investigations in differentiating MET from GBM without surgery.

## 2. Materials and Methods

### 2.1. Dataset and Patient Population

This retrospective study was approved by the Tarbiat Modares University Institutional Review Board, and informed consent from the patients was waived (IR.MODARES.REC.1400.076).

In all cases, the pathology diagnosis was based on WHO standards and was obtained from Hazrate Rasool Akram Hospital, affiliated with Tarbiat Modares University [21]. We have collected MRI data from 91 patients (GBM: 51, MET: 40) based on their pathological confirmation.

Patients with biopsy confirmation of GBM or MET were excluded if they had any of the following conditions:

1. Strokes and infections of the intracranial space
2. The use of antitumor treatments prior to MR scanning, such as brain surgery, chemotherapy, or radiation
3. Inadequate electronic medical records

### 2.2. Image Acquisition

The MR scans were performed using the 1.5T Siemens Trio Scanners in the MR Research Center. In this work, we have concentrated on conventional MR sequences, including T1-weighted imaging (T1WI), contrast-enhanced T1-weighted imaging (T1C), T2-weighted imaging (T2WI), and fluid-attenuated inversion recovery (FLAIR). Patients with intracranial tumors undergo these examinations regularly.

### 2.3. Segmentation and Feature Extraction

All T1WI, T2WI, FLAIR, and T1C images (matrix size:512 × 512, slice thickness = 5 mm, and slice interval = 0 mm) have been transferred from the picture archiving and communication system (PACS) to 3D Slicer [1–6]. Using these images, two radiologists (Reader 1 and 2; 10 years of experience) were blind to grouping manually selected regions of interest (ROIs) along the edge of the tumor. The tumors separately were segmented on all MRI images (T1-weighted imaging (T1WI), contrast-enhanced T1-weighted imaging (T1C), T2-weighted imaging (T2WI), and fluid-attenuated inversion recovery (FLAIR)) to form the volume of interest (VOI). [7–12]. In each slice, ROIs were drawn along the tumor margin to encompass the entire tumor area [14, 17, 22–24]. The preprocessing and feature extraction of the images were performed using Pyradiomics (http://pyradiomics.readthedocs.io/en/latest/index.html) [20, 24–28]. The voxel size resampling (1^∗^1^∗^1) and bin width (64) were applied to the images. Pyradiomics was used to extract radiomic features from each ROI based on its three-dimensional region of interest (3D ROI) [29–34]. From each sequence, 107 features were extracted (Table 1), and these features were grouped into three categories: first-order statistics (*n* = 18), shape-based features (*n* = 14), and textural features. The textural feature category includes GLCM (*n* = 24), GLRLM (*n* = 16), GLSZM (*n* = 16), GLDM (*n* = 14), and NGTDM (*n* = 5) [34–37]. Both the training (70% data) and validation groups (30% data) were normalized using *Z*-scores. Intraobserver and interobserver intraclass correlation coefficients (ICCs) were applied to measure the reproducibility of each feature [18, 19]. Reader 1 and Reader 2 performed image segmentation independently twice weekly to assess intraobserver reliability. Using the following steps, we selected significant radiomic features [18, 19]. ICCs over 0.75 were kept for intraobserver and interobserver features. Following that, LASSO logistic regression was performed with 10-fold cross-validation. In order to generate machine learning inputs, all selected features from all series of images were registered in one row after dimensionality reduction.

The article "Differentiating Glioblastoma Multiforme from Brain Metastases Using Multidimensional Radiomics Features Derived from MRI and Multiple Machine Learning Models" was published in 2022. Journal: Biomed Res Int.

### 2.4. First Radiomics Model Establishment

Eight ML algorithms were imported from the scikit-learn library in Python software to establish models [15, 16, 25, 26, 38]. These algorithms included Support Vector Machine (SVM), Naïve Bayes (NB), Multilayer perceptron (MLP), Decision Tree (DT), Ada Boost (ADA), K-nearest neighbor (K.N.N.), Logistic Regression (LR), and Random Forest (RF) [15, 16, 25, 26, 38].

Selected features from LASSO were imported to this ML, and the predictive ability of each algorithm was primarily assessed using the AUC of receiver operating characteristic (ROC) curve analysis [15, 16, 25, 26, 38].

### 2.5. Second Radiomics Model Establishment (Wavelet-Based Features)

Multidimensional wavelet transforms were created by importing selected features from LASSO. This means that the low pass filter generates the approximate coefficient, and the high pass filter would result in the detail coefficients. The approximate coefficient is the most similar signal to the original signal. The detail coefficient consisted of three matrices: vertical, horizontal, and diagonal [15, 16]. We have considered 31 different wavelet filter banks from four distinct families to provide a wide range of feature vectors from different wavelet filter banks. The 31 different wavelet filter banks “ bior1.3, bior1.5, bior2.2, bior2.4, bior2.6, bior3.1, bior3.3, bior3.5, bior3.7, bior4.4, bior5.5, db2, db3, db4, db5, db6, db7, db8, db9, sym2, sym3, sym4, sym5, sym6, sym7, sym8, coif1, coif2, coif3, coif4, coif5” were among the most conventional filter banks that are available in Python compiler. Features extracted from the 3D Slicer were initially considered as 4-Dimensional signals. These signals were then considered as input signals to multidimensional discrete wavelets. The approximate and detail coefficients were substantially generated and saved in a python array. Approximate coefficients were the most similar signal to the primary signal, and the detail coefficients consisted of horizontal, vertical, and diagonal details (cH1, cV1, cD1). These approximate coefficients and detail coefficients were generated by low and high pass filters, respectively. We calculated eleven different criteria for approximation and detail coefficient matrixes. Seven of these criteria were: maximum, minimum, average, median, standard deviation, Shannon entropy, and signal energy applied to entire approximate coefficient and detail coefficients matrices and led to 28 different feature vectors (7^∗^4). The other two were the standard error and slope between approximate coefficient and detail coefficient matrixes generating six other features (2^∗^3). Eventually, two signal energy and wavelength criteria were used for the whole signal (original input signal), which led to 2 other features and a total of 36 features for every single 3D Slicer output sample. These features were saved in the text file and used as the input file for the machine learning model. These procedures have been done for 31 different wavelet filter banks mentioned earlier, and for each filter bank, we have made a separated feature vectors file. To be more precise, each filter bank had a unique profile; hence, we had 31 different profiles for each sample. Eight ML used these profiles separately as an input file. Finally, we have reported our best result as our proposed model.

The article "Differentiating Glioblastoma Multiforme from Brain Metastases Using Multidimensional Radiomics Features Derived from MRI and Multiple Machine Learning Models" was published in 2022. Journal: Biomed Res Int.

### 2.6. Evaluation Method

Regarding the dataset size, we used the 5-fold cross-validation. To avoid bias, we repeated the 5-fold cross-validation test 100 times. Eventually, the iteration average was considered the model's outputs. The classification influence can be evaluated using three indicators: area under the receiver operating characteristic curve (AUC), accuracy (ACC), and F1-score. Finally, a pairwise test was applied to compare the obtained ROC curves, and the ROC curves of the wide variety of classifiers were then investigated. According to the analysis, *p* < 0.05 illustrates that the two ROC curves were statistically significant differences [20, 24, 25, 38–40]. Workflows are shown in Figures 1 and 2.

## 3. Result

### 3.1. First Radiomics Model Result

We have reported the result of our proposed model by a set of conventional parameters, including F1-score, accuracy, and AUC. These parameters could best express the model's performance in machine learning research. As mentioned in the first model, we have used the selected features obtained from 3D Slicer and used SVM, NB, MLP, DT, ADA, KNN, LR, and RF to establish our predictive model. The highest accuracy for these models is achieved by random forest algorithms, shown in Table 2.

### 3.2. Second Radiomics Model Result

We used the selected feature vector from the 3D Slicer as the multidimensional DWT input for the second model and extracted the approximate and detailed coefficients. After concatenating the approximate coefficient and detail coefficient matrices, particular criteria have been calculated. The same eight ML were applied to establish the predictive model. We calculated accuracy, F1-score, and AUC of ROC in 31 different filter banks, as presented in Tables 3–5.

Our result proved that the second model could perform better than the first model (sig ≤0.05). This model's DB5 filter bank and Logistic Regression achieved the highest result. We have gained 0.98, 0.99, and 0.98 percent for accuracy, AUC-roc, and F1-score, respectively. We introduce the DB5 wavelet and Logistic regression as our proposed model for identifying the GBM and MET in MRI sequences. These differences are shown in Tables 6–8.

## 4. Discussion

We explored the diagnostic performance of radiomics using traditional machine learning classifiers for differentiating GBM from single MET. The wavelet radiomics performed better than the best-performing traditional radiomics and demonstrated good generalizability in the testing data. Four imaging modes were used, 107 features were extracted from each sequence, and all 428 parameters were used as LASSO inputs to select the best features. The selected features are used in two different ways. First, used in ML input, then transferred to 31 wavelet filter banks, and lastly imputed to ML. For the best combination of classification procedures, extensive comparative studies were performed for 31 types of wavelet features and eight classification algorithms (Adaboost, K.N.N., Gaussian NB, DT, LR, SVM, RF, and MLP).

The article "Differentiating Glioblastoma Multiforme from Brain Metastases Using Multidimensional Radiomics Features Derived from MRI and Multiple Machine Learning Models" was published in 2022. Journal: Biomed Res Int.

Moreover, the multidimensional discrete wavelet could reveal the hidden feature of the data. Multidimensional discrete wavelets provide us with approximate and detailed coefficient matrices. The approximate coefficient is the most similar wave to the original signal, while the detailed coefficient includes horizontal, vertical, and diagonal details. We found that wavelet feature extraction, a critical classification component, enables us to distinguish different tumor characteristics using different feature types.

According to our findings, wavelet radiomics-based ML can successfully discriminate GBM and MET. LR was judged to be the most effective model. Another important finding from our research was the diagnostic performance of the top models with wavelet features outperformed models without wavelet features (Tables 6–8).

Our study's most important outcome was identifying appropriate discriminative models for lesions in the brain. LR (AUC 0.99) and RF (AUC 0.97) are both high-performing models for GBM and MET classification.

A number of previous studies have used multiparametric MRI data to discriminate between GBM tumors and MET, including advanced imaging methods such as diffusion, perfusion, and MR spectroscopy [1–6]. It should be noted that advanced imaging is not incorporated into all MRI protocols across all sites and is highly dependent on the acquisition and analysis method [14, 34, 41]. Therefore, it is important to be able to classify brain tumors based on common sequences [14, 34, 41]. Some previous studies attempted to distinguish between different types of brain tumors based on a single contrast; however, these studies were carried out on relatively small populations and were limited to data obtained from a specific MRI system [14, 34].

Cho1 et al. [42] studied radiomics and ML in glioma grading classification, which showed that RF and LR were high-performing models. In our investigation, the LR model with db5 wavelet feature performed better (AUC 0.99) than the LR model in a previous study by Cho et al., which had an AUC of 0.95. These findings demonstrate that the proposed model has an impact on model performance. Our results were better than the previous study that looked at various ML. Priya et al. [22] used the LASOO and Elastic Net model to classify brain tumors; we have higher results in wavelet base feature (0.99 vs. 095) and worse in part without wavelet base features (0.95 vs. 0.93).

The article "Differentiating Glioblastoma Multiforme from Brain Metastases Using Multidimensional Radiomics Features Derived from MRI and Multiple Machine Learning Models" was published in 2022. Journal: Biomed Res Int.

Ning et al. [43] examined seven ML classifiers and five feature reduction techniques using radiomics features produced from T1-CE and T2W pictures and obtained an AUC of 0.890 with an accuracy of 83 percent. The second part of their work used deep neural networks, which had an AUC of 0.95 and an accuracy of 89%. Even though we did not analyze deep neural networks (DNN) due to their computational cost, our findings were comparable to Ning et al.

Su et al. [17] extracted features from the T1-CE sequence, then evaluating 30 model combinations and feature reduction for their radiomics obtained an AUC of 0.80. Using 248 combinations of wavelet feature series and classifier, we achieved a higher AUC of 0.99 and an accuracy of 98 percent. The fact that we extracted wavelet features from MRI sequences improved our results.

Wavelet feature is an essential element of this model performance. The improved effectiveness of 31 types of wavelet features compared to a priori feature (without wavelet) was a key conclusion of our research. LR and RF models provide a more significant generalizability benefit than other ML models. We have found the essential type of wavelets for Ada, Knn, Nb, Dt, LR, SVM, RF, and MLP were db8, coif2, bior2.6, bior1.5, db5, db2, bior1.5, and coif3 consequently.

Adding wavelets to the analysis confirms that it can better distinguish MET and GBM than the radiomics model based solely on c MRI features. Therefore, our study provides a good solution to the problem of poor model performance in radiomics research. We propose a unique, helpful prediction model based on MRI sequences (T1-W, T2-W, T1C-W, and Flair-W) that can be used in clinical practice.

### 4.1. Limitation

Our research has a few limitations that need to be addressed. First, due to the retrospective nature of the investigation, several patients' clinical information and MRI sequences were missing, resulting in a smaller sample size. Second, although normalization was implemented during data preprocessing, variation across MRI scan protocols was unavoidable. Third, the picture segmentation approach utilized in this work relied on manual delineation, which might be replaced by automated delineation of ROIs using deep learning methods in the future to enhance the model's reliability. Fourth, since our conclusion that radiomics characteristics may represent changes in the tumor microenvironment was based on circumstantial evidence, further validation and experimental confirmation are required. Finally, our study did not include advanced sequences, such as DWI or perfusion MR imaging.

The article "Differentiating Glioblastoma Multiforme from Brain Metastases Using Multidimensional Radiomics Features Derived from MRI and Multiple Machine Learning Models" was published in 2022. Journal: Biomed Res Int.

## 5. Conclusion

We found that radiomics-based ML can accurately classify GBM and MET. Also, in this study, the best results were in the LR algorithm and wavelet db5, which can be considered acceptable in data with few samples. The performance of a model might vary based on the mix of classifier and feature types used. Thus a complete model selection method should be used. Also, the result of the models applied to the extracted features' composition is very suitable compared to their separate modes.

## Figures and Tables

**Figure 1:** Flowchart of the process of radiomics. The tumors were segmented on all MRI images to form the volume of interest (VOI). The machine learning algorithm was then used to fit the best predictive model.

**Figure 2:** Flowchart of the process of wavelet radiomics. The tumors were segmented on all MRI images to form the volume of interest (VOI). Different filter banks are applied to them and the machine learning algorithm was used to fit the best predictive model.

**Table 1:** Feature extracted from the 3D Slicer.

Feature groups	Feature type
Shape features	Elongation, Flatness, LeastAxisLength, MajorAxisLength, Maximum2DDiameterColumn, Maximum2DDiameterRow, Maximum2DDiameterSlice, Maximum3DDiameter, MeshVolume, MinorAxisLength, Sphericity, SurfaceArea, SurfaceVolumeRatio, VoxelVolume
First-order statistics	10Percentile, 90Percentile, Energy, Entropy, InterquartileRange, Kurtosis, Maximum, MeanAbsoluteDeviation, Mean, Median, Minimum, Range, RobustMeanAbsoluteDeviation, RootMeanSquared, Skewness, TotalEnergy, Uniformity, Variance
Gray-level dependence matrix (GLDM)	DependenceEntropy, DependenceNonUniformity, DependenceNonUniformityNormalized, DependenceVariance, GrayLevelNonUniformity, GrayLevelVariance, HighGrayLevelEmphasis, LargeDependenceEmphasis, LargeDependenceHighGrayLevelEmphasis, LargeDependenceLowGrayLevelEmphasis, LowGrayLevelEmphasis, SmallDependenceEmphasis, SmallDependenceHighGrayLevelEmphasis, SmallDependenceLowGrayLevelEmphasis
Gray-level run length matrix (GLRLM)	GrayLevelNonUniformity, GrayLevelNonUniformityNormalized, GrayLevelVariance, HighGrayLevelRunEmphasis, LongRunEmphasis, LongRunHighGrayLevelEmphasis, LongRunLowGrayLevelEmphasis, LowGrayLevelRunEmphasis, RunEntropy, RunLengthNonUniformity, RunLengthNonUniformityNormalized, RunPercentage, RunVariance, ShortRunEmphasis, ShortRunHighGrayLevelEmphasis, ShortRunLowGrayLevelEmphasis
Gray-level cooccurrence matrix (GLCM)	Autocorrelation, ClusterProminence, ClusterShade, ClusterTendency, Contrast, Correlation, DifferenceAverage, DifferenceEntropy, DifferenceVariance, inverse difference (ID), inverse difference moment (IDM), inverse difference moment normalized (IDMN), inverse difference normalized (IDN), informal measure of correlation (IMC) 1, informal measure of correlation (IMC) 2, InverseVariance, JointAverage, JointEnergy, JointEntropy, MCC, MaximumProbability, SumAverage, SumEntropy, SumSquares
Gray-level size-zone matrix (GLSZM)	GrayLevelNonUniformity, GrayLevelNonUniformityNormalized, GrayLevelVariance, HighGrayLevelZoneEmphasis, LargeAreaEmphasis, LargeAreaHighGrayLevelEmphasis, LargeAreaLowGrayLevelEmphasis, LowGrayLevelZoneEmphasis, SizeZoneNonUniformity, SizeZoneNonUniformityNormalized, SmallAreaEmphasis, SmallAreaHighGrayLevelEmphasis, SmallAreaLowGrayLevelEmphasis, ZoneEntropy, ZonePercentage, ZoneVariance
Neighboring gray tone difference matrix (NGTDM)	Busyness, Coarseness, Complexity, Contrast, Strength

The article "Differentiating Glioblastoma Multiforme from Brain Metastases Using Multidimensional Radiomics Features Derived from MRI and Multiple Machine Learning Models" was published in 2022. Journal: Biomed Res Int.

**Table 2:** Performance models in test data (feature without wavelet).

Models	Accuracy	AUC	F1-score
MLP	0.90	0.90	0.90
RF	0.92	0.94	0.94
SVM	0.57	0.55	0.71
LR	0.93	0.88	0.90
DT	0.91	0.92	0.91
Nb	0.64	0.86	0.52
Knn	0.79	0.90	0.79
Ada	0.90	0.92	0.91

**Table 3:** Accuracy in 31 different filter banks.

	Ada	Knn	Nb	Dt	LR	SVM	RF	MLP
bior1.3	0.933189	0.891721	0.61068	0.905832	0.941758	0.912761	0.945032	0.950985
bior1.5	0.965257	0.94742	0.646329	0.914328	0.956465	0.832176	0.973847	0.947466
bior2.2	0.923965	0.866087	0.645475	0.899008	0.924443	0.704708	0.94095	0.907554
bior2.4	0.94369	0.90734	0.695714	0.912643	0.948408	0.777932	0.942614	0.922503
bior2.6	0.95082	0.920852	0.693796	0.886444	0.931135	0.767052	0.952591	0.947212
bior3.1	0.927787	0.907053	0.60877	0.880337	0.893043	0.799389	0.958945	0.909473
bior3.3	0.925133	0.943487	0.656289	0.876967	0.953993	0.796909	0.968925	0.932868
bior3.5	0.930002	0.936131	0.604197	0.903743	0.947655	0.792489	0.944739	0.950133
bior3.7	0.927571	0.943129	0.634732	0.886911	0.948263	0.799461	0.945879	0.93021
bior4.4	0.93232	0.95518	0.62868	0.917023	0.938454	0.797078	0.947979	0.947715
bior5.5	0.933369	0.941989	0.612398	0.906204	0.934667	0.801717	0.956616	0.954862
coif1	0.922405	0.902193	0.608189	0.89412	0.930878	0.872911	0.946356	0.962986
coif2	0.943946	0.955792	0.635985	0.900505	0.958749	0.813401	0.954382	0.948507
coif3	0.9467	0.945316	0.629187	0.900545	0.964684	0.889525	0.952297	0.964193
coif4	0.920573	0.927746	0.61435	0.883489	0.946937	0.934528	0.964741	0.958771
coif5	0.944292	0.875767	0.599845	0.869593	0.898315	0.865067	0.959446	0.927132
db2	0.928196	0.903953	0.588558	0.849616	0.932377	0.950546	0.950244	0.940636
db3	0.918309	0.942918	0.631876	0.873505	0.907149	0.746167	0.947854	0.936909
db4	0.932921	0.926325	0.632563	0.892192	0.939004	0.776472	0.937961	0.916678
db5	0.926129	0.941244	0.619148	0.923357	0.988745	0.796044	0.951191	0.952799
db6	0.936539	0.951273	0.616145	0.904428	0.932609	0.806208	0.941486	0.939429
db7	0.922993	0.953972	0.643097	0.893853	0.954054	0.818546	0.959917	0.953336
db8	0.95857	0.929108	0.642418	0.90545	0.938197	0.863222	0.969784	0.929326
db9	0.924636	0.944797	0.645315	0.875302	0.929999	0.945966	0.969645	0.935359
sym2	0.933876	0.893567	0.565925	0.850802	0.933613	0.920392	0.946448	0.939357
sym3	0.916029	0.943786	0.628778	0.871188	0.936641	0.810063	0.946932	0.930468
sym4	0.947051	0.953057	0.655627	0.903845	0.948039	0.845584	0.956469	0.9603
sym5	0.933549	0.919176	0.647675	0.896683	0.928433	0.806217	0.954992	0.910095
sym6	0.933247	0.947034	0.636997	0.88298	0.936826	0.815107	0.943306	0.910482
sym7	0.942203	0.94351	0.634277	0.901731	0.967642	0.825141	0.959545	0.952585
sym8	0.922269	0.924227	0.647042	0.886828	0.925618	0.805148	0.951747	0.907678

The article "Differentiating Glioblastoma Multiforme from Brain Metastases Using Multidimensional Radiomics Features Derived from MRI and Multiple Machine Learning Models" was published in 2022. Journal: Biomed Res Int.

**Table 4:** F1-score in 31 different filter banks.

	Ada	Knn	Nb	Dt	LR	SVM	RF	MLP
bior1.3	0.933189	0.891721	0.61068	0.905832	0.941758	0.912761	0.945032	0.950985
bior1.5	0.965257	0.94742	0.646329	0.914328	0.956465	0.832176	0.973847	0.947466
bior2.2	0.923965	0.866087	0.645475	0.899008	0.924443	0.704708	0.94095	0.907554
bior2.4	0.94369	0.90734	0.695714	0.912643	0.948408	0.777932	0.942614	0.922503
bior2.6	0.95082	0.920852	0.693796	0.886444	0.931135	0.767052	0.952591	0.947212
bior3.1	0.927787	0.907053	0.60877	0.880337	0.893043	0.799389	0.958945	0.909473
bior3.3	0.925133	0.943487	0.656289	0.876967	0.953993	0.796909	0.968925	0.932868
bior3.5	0.930002	0.936131	0.604197	0.903743	0.947655	0.792489	0.944739	0.950133
bior3.7	0.927571	0.943129	0.634732	0.886911	0.948263	0.799461	0.945879	0.93021
bior4.4	0.93232	0.95518	0.62868	0.917023	0.938454	0.797078	0.947979	0.947715
bior5.5	0.933369	0.941989	0.612398	0.906204	0.934667	0.801717	0.956616	0.954862
coif1	0.922405	0.902193	0.608189	0.89412	0.930878	0.872911	0.946356	0.962986
coif2	0.943946	0.955792	0.635985	0.900505	0.958749	0.813401	0.954382	0.948507
coif3	0.9467	0.945316	0.629187	0.900545	0.964684	0.889525	0.952297	0.964193
coif4	0.920573	0.927746	0.61435	0.883489	0.946937	0.934528	0.964741	0.958771
coif5	0.944292	0.875767	0.599845	0.869593	0.898315	0.865067	0.959446	0.927132
db2	0.928196	0.903953	0.588558	0.849616	0.932377	0.950546	0.950244	0.940636
db3	0.918309	0.942918	0.631876	0.873505	0.907149	0.746167	0.947854	0.936909
db4	0.932921	0.926325	0.632563	0.892192	0.939004	0.776472	0.937961	0.916678
db5	0.926129	0.941244	0.619148	0.923357	0.988745	0.796044	0.951191	0.952799
db6	0.936539	0.951273	0.616145	0.904428	0.932609	0.806208	0.941486	0.939429
db7	0.922993	0.953972	0.643097	0.893853	0.954054	0.818546	0.959917	0.953336
db8	0.95857	0.929108	0.642418	0.90545	0.938197	0.863222	0.969784	0.929326
db9	0.924636	0.944797	0.645315	0.875302	0.929999	0.945966	0.969645	0.935359
sym2	0.933876	0.893567	0.565925	0.850802	0.933613	0.920392	0.946448	0.939357
sym3	0.916029	0.943786	0.628778	0.871188	0.936641	0.810063	0.946932	0.930468
sym4	0.947051	0.953057	0.655627	0.903845	0.948039	0.845584	0.956469	0.9603
sym5	0.933549	0.919176	0.647675	0.896683	0.928433	0.806217	0.954992	0.910095
sym6	0.933247	0.947034	0.636997	0.88298	0.936826	0.815107	0.943306	0.910482
sym7	0.942203	0.94351	0.634277	0.901731	0.967642	0.825141	0.959545	0.952585
sym8	0.922269	0.924227	0.647042	0.886828	0.925618	0.805148	0.951747	0.907678

The article "Differentiating Glioblastoma Multiforme from Brain Metastases Using Multidimensional Radiomics Features Derived from MRI and Multiple Machine Learning Models" was published in 2022. Journal: Biomed Res Int.

**Table 5:** AUC of ROC in 31 different filter banks.

	Ada	Knn	Nb	Dt	LR	SVM	RF	MLP
bior1.3	0.936	0.900667	0.670833	0.9075	0.946	0.920833	0.947167	0.955333
bior1.5	0.968417	0.950083	0.715833	0.92325	0.95825	0.8265	0.975583	0.9505
bior2.2	0.927417	0.881417	0.694417	0.903667	0.927833	0.563917	0.942	0.912833
bior2.4	0.9445	0.916083	0.74525	0.912833	0.949167	0.753333	0.9425	0.925083
bior2.6	0.95275	0.93025	0.747333	0.890833	0.93675	0.757083	0.952	0.950083
bior3.1	0.93375	0.911583	0.658083	0.886417	0.895333	0.809167	0.959	0.913417
bior3.3	0.93	0.947667	0.71075	0.87775	0.959417	0.784583	0.969333	0.936583
bior3.5	0.93325	0.938917	0.669167	0.904333	0.952667	0.779583	0.94325	0.952833
bior3.7	0.933083	0.946833	0.6945	0.888	0.9525	0.784167	0.946667	0.933167
bior4.4	0.9355	0.9555	0.68875	0.914917	0.938917	0.776917	0.947417	0.94925
bior5.5	0.938	0.940917	0.683917	0.905417	0.937167	0.786833	0.95575	0.95675
coif1	0.928	0.904917	0.673167	0.896667	0.930333	0.881	0.948667	0.964
coif2	0.944833	0.960417	0.694583	0.89725	0.95975	0.799167	0.95275	0.950417
coif3	0.9485	0.945833	0.690417	0.9005	0.9625	0.883333	0.950583	0.96375
coif4	0.924167	0.933417	0.670917	0.891333	0.949833	0.93825	0.964583	0.958917
coif5	0.9485	0.87825	0.660833	0.876083	0.901667	0.879417	0.959167	0.927667
db2	0.933417	0.913583	0.637167	0.855167	0.933833	0.955667	0.95225	0.9435
db3	0.920917	0.94925	0.690417	0.878083	0.91175	0.707583	0.948917	0.937833
db4	0.93575	0.92925	0.69525	0.889333	0.943	0.765	0.93825	0.921583
db5	0.927667	0.941583	0.68125	0.920833	0.991333	0.779167	0.949	0.954667
db6	0.939333	0.948167	0.681	0.903	0.932833	0.79375	0.94175	0.938
db7	0.927	0.955083	0.711167	0.894417	0.952583	0.806917	0.958417	0.952417
db8	0.961833	0.931917	0.700083	0.90575	0.939	0.862583	0.970583	0.931833
db9	0.929083	0.945333	0.7005	0.878667	0.929583	0.944083	0.969167	0.934583
sym2	0.938667	0.89875	0.626667	0.85375	0.935667	0.92275	0.949583	0.940333
sym3	0.917583	0.951583	0.6835	0.875917	0.940333	0.806917	0.949917	0.9325
sym4	0.950083	0.957833	0.7125	0.909167	0.950417	0.8325	0.953833	0.96075
sym5	0.937167	0.921917	0.702833	0.895917	0.933167	0.785833	0.9555	0.913667
sym6	0.938417	0.950417	0.700667	0.886167	0.935667	0.803667	0.941583	0.912917
sym7	0.944	0.945167	0.698083	0.902083	0.967333	0.806667	0.957917	0.9535
sym8	0.925417	0.928167	0.709	0.89	0.928167	0.783	0.950417	0.910083

The article "Differentiating Glioblastoma Multiforme from Brain Metastases Using Multidimensional Radiomics Features Derived from MRI and Multiple Machine Learning Models" was published in 2022. Journal: Biomed Res Int.

**Table 6:** Comparing AUC in the first and second model.

Best results of models	Ada	Knn	Nb	Dt	LR	SVM	RF	MLP
Wavelet type	bior1.5 0.97	coif2 0.96	bior2.6 0.75	bior1.5 0.92	db5 0.99	db2 0.96	db8 0.97	coif1 0.96
Without wavelet	0.92	0.90	0.86	0.92	0.88	0.55	0.94	0.90
%increase (significant: ^∗∗^, no significance ^∗^)	+5.5%^∗∗^	+6.6%^∗∗^	-12.7%^∗∗^	0^∗^	+12.5%^∗∗^	+74.5%^∗∗^	3.19^∗^	6.6%^∗∗^

**Table 7:** Comparing accuracy in the first and second model.

Best results of models	Ada	Knn	Nb	Dt	LR	SVM	RF	MLP
Wavelet type	db8 0.96	coif2 0.96	bior2.6 0.70	bior1.5 0.92	db5 0.99	db2 0.95	bior1.5 0.97	coif3 0.96
Without wavelet	0.90	0.79	0.64	0.91	0.94	0.57	0.92	0.90
%increase (significant: ^∗∗^, no significance ^∗^)	+%6.6^∗∗^	+%21.5^∗∗^	+%9.3^∗∗^	+%1^∗^	+%5.3^∗∗^	+%66.6^∗∗^	+%3^∗^	+%6.6^∗∗^

**Table 8:** Comparing F1-score in the first and second model.

Best results of models	Ada	Knn	Nb	Dt	LR	SVM	RF	MLP
Wavelet type	bior1.5 0.96	coif2 0.96	bior2.4 0.69	db5 0.92	db5 0.99	db2 0.95	bior1.5 0.97	coif3 0.96
Without wavelet	0.91	0.79	0.52	0.91	0.90	0.71	0.94	0.90
% increase (significant: ^∗∗^, no significance ^∗^)	+%5.5^∗∗^	+%21.5^∗∗^	+%32^∗∗^	+%1^∗^	+%10^∗∗^	+%33.82^∗∗^	+%3.19^∗^	+%6.6^∗∗^

## Data Availability

The datasets used and/or analyzed during the current study are available from the corresponding author on reasonable request.
